# Targeting PI3K in cancer: mechanisms and advances in clinical trials

**DOI:** 10.1186/s12943-019-0954-x

**Published:** 2019-02-19

**Authors:** Jing Yang, Ji Nie, Xuelei Ma, Yuquan Wei, Yong Peng, Xiawei Wei

**Affiliations:** Laboratory of Aging Research and Cancer Drug Target, State Key Laboratory of Biotherapy and Cancer Center, National Clinical Research Center for Geriatrics, West China Hospital, Sichuan University, Chengdu, 610041 Sichuan China

**Keywords:** PI3K, mTOR, Cancer, Target therapy

## Abstract

Phosphatidylinositol-3-kinase (PI3K)/AKT/mammalian target of rapamycin (mTOR) signaling is one of the most important intracellular pathways, which can be considered as a master regulator for cancer. Enormous efforts have been dedicated to the development of drugs targeting PI3K signaling, many of which are currently employed in clinical trials evaluation, and it is becoming increasingly clear that PI3K inhibitors are effective in inhibiting tumor progression. PI3K inhibitors are subdivided into dual PI3K/mTOR inhibitors, pan-PI3K inhibitors and isoform-specific inhibitors. In this review, we performed a critical review to summarize the role of the PI3K pathway in tumor development, recent PI3K inhibitors development based on clinical trials, and the mechanisms of resistance to PI3K inhibition.

## Highlights

Activation of the PI3K pathway contributes to the development of tumor PI3K is an attractive therapeutic direction in the treatment of cancer. Inhibition of PI3K signaling is effective in the treatment of several types of cancer. Intrinsic and acquired resistance limits the therapeutic efficacy of PI3K inhibitors.

## Introduction

Phosphatidylinositol-3-kinase (PI3K)/AKT/mammalian target of rapamycin (mTOR) signaling is one of the most important intracellular pathways, which regulates cell growth, motility, survival, metabolism, and angiogenesis [1, 2]. Activation of the PI3K/AKT/mTOR pathway contributes to the development of tumor and resistance to anticancer therapies [3]. MicroRNA (miRNA) and long non-coding RNA (lncRNA), the two most studied classes of non-coding RNA (ncRNA), are crucial regulators of gene expression [4]. These two types of ncRNA and PI3K/AKT/mTOR pathway are in tight conjunction during oncogenesis [5, 6]. The PI3K/AKT/mTOR pathway has been found to be dysregulated almost in all human cancers, such as breast cancer, colorectal cancer, and hematologic malignancies, which emphasizes the value of targeting this pathway as a potential therapeutic direction in the treatment of cancer [7]. Inhibition of PI3K can result in both decreased cellular proliferation and increased cellular death [8]. Small molecule inhibitors of PI3K include PI3K/mTOR inhibitors, pan-PI3K inhibitors, and isoform-selective PI3K inhibitors. The safety and efficacy of these therapeutic approaches have been investigated in a wide range of preclinical and clinical trials, and it is becoming increasingly clear that PI3K inhibitors are effective in inhibiting tumor progression. For example, PI3K delta-specific inhibitor idelalisib is the first PI3Ki compound approved by United States Food and Drug Administration (FDA) and is proved to be effective in the cancer treatment [9]. In this review, we summarized the role of the PI3K signaling in tumor progression, recent PI3K inhibitors development based on clinical trials, and the mechanisms of resistance to PI3K inhibition.

## PI3K signal pathway

### Signal transduction pathways

PI3K is a group of plasma membrane-associated lipid kinases, consisting of three subunits: p85 regulatory subunit, p55 regulatory subunit, and p110 catalytic subunit [10]. According to their different structures and specific substrates, PI3K is divided into 3 classes: classes I, II, and III [1, 2]. Class I PI3Ks comprised of class IA and class IB PI3Ks. Class IA PI3K, a heterodimer of p58 regulatory subunit and p110 catalytic subunit, is the type most clearly implicated in human cancer [11]. Class IA PI3K contains p110α, p110β and p110δ catalytic subunits produced from different genes (PIK3CA, PIK3CB and PIK3CD, respectively), while p110γ produced by PIK3CG represents the only catalytic subunit in class IB PI3K [12]. The p85 regulatory subunit is composed of p85a (p85a, p55a and p50a splice variants), p85b and p55g, which are encoded by the genes PIK3R1, PIK3R2 and PIK3R3, respectively [2]. As an integration point for p110 activation and downstream molecular, p85 regulatory subunit binds and integrates signals from various transmembrane and intracellular proteins, including tyrosine kinase-linked receptors, protein kinase C (PKC), Src homology 2 domain-containing protein tyrosine phosphatase 1 (SHP1), Rac, Rho, hormonal receptors, Src, as well as mutated Ras [8]. The overview of PI3K/AKT/mTOR signaling pathway was shown in Fig. 1.

**Fig. 1:** The overview of PI3K/AKT/mTOR signaling pathway

### Activation of PI3K signaling

Under baseline conditions, the p110 catalytic subunit is stabilized by dimerization with regulatory p85 subunit. In physiologic conditions, PI3K is normally activated by a variety of extracellular stimuli, such as growth factors, cytokines, and hormones [13]. Upon activation, PI3K catalyzes the phosphorylation of PtdIns(4,5) P2(PIP2) to produce PtdIns(3,4,5) P3(PIP3), a second messenger that binds and recruits a subset of pleckstrin-homology (PH), FYVE, Phox (PX), C1, C2 or other lipid-binding domains of downstream targets to the cell membrane. A variety of signaling proteins, such as kinases AKT and PDK1 can bind to the lipid products of PI3K and thereby localize to the cell membrane to activate cell growth and cell survival pathways [14]. Phosphatase and tensin homologue deleted on chromosome 10 (PTEN) regulates the pathway by dephosphorylating PIP3 to PIP2 and thus prevents activation of downstream kinases [8].

In the last decade or so, ncRNAs have emerged as important regulators of a wide range of genes and PI3K/AKT/mTOR pathway [5, 6]. ncRNAs function as both upstream mediators and downstream effectors to affect PI3K pathway activities. Of importance, ncRNAs have been reported to directly or indirectly target multiple key components (PI3K, AKT, mTOR and PTEN) in the PI3K pathway, regulating the activity of PI3K signaling. However, the exact mechanisms through which lncRNAs directly or indirectly affect PI3K have not been fully studied.

## PI3K signaling in human cancer

Over the past decades, PI3K signaling pathway is believed to be deregulated in a wide spectrum of human cancers. Mutations of the kinases and/or decreased expression of PTEN lead to neoplastic transformation, underscoring its central role in human carcinogenesis [8, 15]. PI3K pathway is deregulated through a variety of mechanisms, including loss or inactivation of the tumor suppressor PTEN, mutation or amplification of PI3K, as well as activation of tyrosine kinase growth factor receptors or oncogenes upstream of PI3K [16–18].

### Loss or inactivation of PTEN

PTEN, a negative regulator of PI3K pathway, acts as a direct antagonist of PI3K action through dephosphorylation of PIP3. Dimeric PTEN complexes have higher activity than PTEN monomers in PIP3 dephosphorylation and PI3K signaling regulation [19, 20]. PTEN is a well characterized tumor suppressor with growth, survival and metabolic regulatory functions, and its loss or inactivation of function is frequently observed in both heritable and sporadic malignances, including brain cancer, breast cancer, and prostate cancer [21–23]. Furthermore, it has been shown that small changes in PTEN expression contribute to major consequences for normal cellular function [24]. In PTEN knock-in mice harboring two cancer-associated PTEN mutations, PTENC124S and PTENG129E inhibit the PTEN lipid-phosphatase activity in a dominant negative manner, leading to increased activity of PI3K signaling and tumorigenesis [20]. Moreover, in PTEN-deficient cancer, the main carcinogenic driving force is the overactivation of AKT caused by the loss of PTEN lipid phosphatase function [20, 25].

### Mutation or amplification of PI3K

PIK3CA (phosphatidylinositol 3-kinase, catalytic, α-polypeptide), the gene encoding the p110α subunit, are frequently mutated or amplified in the most common human cancers, such as breast cancers, colon cancer, gastric cancer, cervical cancer, prostate cancer, and lung cancer [26–31]. Most mutations cluster around two hotspots: E545K (exon 9) in the helical phosphatidylinositol kinase homology domain, which reduces inhibition of p110α by the regulatory subunit p85; H1047 (exon 20) near the end of the catalytic domain, which increases interaction of p110α with lipid membranes [32, 33]. E542K is also one of the most frequently observed PIK3CA mutations [33, 34]. In colorectal cancer, exon 9 plays a more important role than exon 20, whereas in endometrial cancer, the opposite pattern was described, suggesting that different mutations of PIK3CA may have specific effects on downstream carcinogenic signals [35]. It is worth noting that the coexistence of mutations in helical domain and kinase domain leads to synergistic enhancement of p110 activity and enhancement of the tumorigenicity effects [35]. In addition to the two hotspot mutations, mutations on C2 domain are also important components of PIK3CA mutations [36]. Such deregulation of PI3K pathway promotes cell proliferation and migration, glucose transport and catabolism, cytoskeletal rearrangements, and angiogenesis, playing an important role in tumor initiation, progression, and maintenance [27]. In addition, the tumorigenic potential of these mutations was confirmed in experimental research using genetically engineered mouse models (GEMMs) [37–39].

In contrast, mutations in the other catalytic subunits p110β, p110γ and p110δ are rare, and overexpression of these wild-type catalytic subunits is sufficient to induce an oncogenic phenotype in cultured cells [34, 40]. Subunit p110β plays an important role in stimulating cell proliferation, invasiveness, as well as tumorigenesis in prostate and breast cancer [41–43]. The precise mechanisms of p110β activation in cancer are still not well established. However, it has been reported that it can occur through G protein-coupled receptor (GPCRs) [44]. E633K, a p110β helical domain mutation, was first reported in a HER2-positive breast cancer patient [45]. E633K might enhance p110β’s basal association with membranes and thus activates p110β [43]. The p110β has been suggested to be responsible for the reaccumulation of PIP3 and reactivation of AKT in HER2-amplified cancers treated with a p110α-specific inhibitor, and concomitant inhibition of p110α and p110β induces greater antitumor efficacy in HER2-amplified and PIK3CA mutant breast cancers. In endometrial cancer, occurrence of PIK3CB mutations (D1067V and A1048V within the kinase domain) has been reported [46, 47]. PI3Kδ is primarily expressed in the cells of hematopoietic lineage and is activated by cytokine receptors, antigen receptors, growth factor receptors and costimulatory receptors [48, 49]. PI3Kδ is important in T and B cells development and activation. PI3Kδ blockade increases genomic instability by an activation-induced cytidine deaminase (AID)-dependent mechanism in B cells [50]. Gain-of-function (GOF) mutations in PI3Kδ result in a range of developmental and functional deficiencies of B and T cell that compromise host defense. Loss-of-function (LOF) mutations lead to much more severe B cell lymphopenia and agammaglobulinemia, but not T cell senescence [51]. In acute myeloid leukemia (AML), PI3Kδ is critical in activation of AKT and cell proliferation [52]. Point mutations of p110δ have been described in a panel of diffuse large B-cell lymphomas [53]. Moreover, p110δ protein has been detected in cells of melanocytic or breast origin and it has been reported to regulate cell migration in breast cancer lines and tumor progression [54]. PI3Kγ is abundantly expressed in immune cells of myeloid origin but not cancer cells, which regulates innate immunity in both inflammation and cancer [55]. P110γ contributes to chemotactic responses, as well as reactive oxygen species production in neutrophils [56]. PI3Kγ may possibly be able to promote solid tumor neovascularization indirectly by regulating the immune-suppressive TAM subset, which is a major source of VEGFα [57].

### Non-coding RNA and other factors in regulation of PI3K pathway

In addition to inherent aberrations in members of the PI3K pathway, pathologic signaling through this pathway can also occur in other ways, including tyrosine kinase growth factor receptors (e.g. human epidermal growth factor receptor 2 and insulin-like growth factor − 1 receptor), cell adhesion molecules (e.g. integrins, GPCR), and oncogenes (e.g. RAS) [1, 58, 59]. The interactions between ncRNAs and PI3K signaling in cancer have been studied. For example, the lncRNA CRNDE which promote cell proliferation through activating PI3K signaling, is highly expressed in patients with non-small cell lung cancer, colorectal cancer, gastric cancer, cervical cancer, heptaocellular carcinoma and gallbladder cancer [60–65]. In addition to activating PI3K pathway, some ncRNAs have been reported to inhibit the activity of PI3K signaling. lncRNA GAS5 expression is lower in tumor cells compared to normal cells; its over-expression inhibits tumor cell proliferation and migration while treatment with PI3K activator reduces the inhibitory effects [66–72]. Table 1 shows the examples of lncRNA that interact with PI3K signaling in different types of cancer.

**Table 1:** Important long non-coding RNA that interact with PI3K signaling in different cancer

LncRNAs	Up- or down-regulation	Cancer type	Affected biological process (Involved factors)	References
CRNDE	Up	Gallbladder carcinoma; Non-small cell lung carcinoma; Colorectal cancer; Gastric cancer; Cervical cancer; Heptaocellular cancer	Cell roliferation, growth, migration, invasion and apoptosis; glucose and lipid metabolism (Gene expression in PI3K pathway: MMP-9, JUK-1, ERK and AKT)	[60–65]
OIP5-AS1	Up	Multiple myeloma; Osteosarcoma	Cell proliferation, cycle and apoptosis; cisplatin resistance, (miRNA-410, miRNA-340-5p and expression of lysophosphatidic acid acyltransferase)	[201, 213]
CCAT1	Up	Thyroid carcinoma; Squamous cell carcinomas	Cell proliferation, migration, and invasion (miRNA-143; EGFR expression)	[214, 215]
H19	Up	Retinoblastoma, Melanoma	Cell viability, migration, invasion, and apoptosis (miRNA-143, RUNX2, Phosphorylation of key kinases)	[216, 217]
HOTAIR	UP	Gastric cancer; Adenocarcinoma of esophagogastric junction; Leukemia; Melanoma; Gliomas	Cell proliferation, metastasis and apoptosis; cisplatin resistance; acquired multidrug resistance to imatinib (miRNA-143, miRNA-34a, miRNA-152-3p, miRNA-126, miRNA-326, FGF1)	[202, 203, 218–222]
NEAT1	Up	Myeloma; Cervical carcinoma; Gastric cancer	Cell proliferation, viability, migration, invasion, apoptosis, and cell cycle. (microRNA-17)	[223–226]
HULC	Up	Bladder cancer; Leukemia; Gliomas; Osteosarcoma; Liver cancer; Gastric cancer	Cell viability, growth, migration, invasion and autophagy (PTEN, miRNA15a, autophagy-P62, miRNA-122)	[227–232]
AB073614	Up	Colorectal cancer	Cell cycle, proliferation, migration, and invasion	[233]
PTTG3P	Up	Hepatocellular carcinoma	Cell proliferation, migration, invasion, tumorigenesis and metastasis	[234]
MALAT1	Up	Cervical cancer; Epithelial ovarian cancer; Breast cancer; Osteosarcoma; Cholangiocarcinoma; Non-small cell lung carcinoma; Hepatocellular carcinoma; Renal cell carcinoma	Cell proliferation, invasion, metastasis, viability and mobility; stemness-related factor activation; epithelial-to-mesenchymal transition; cisplatin resistance (PI3Kp85α, miRNA-22-3p, miRNA195, miRNA-124, MiRNA-101-3p, miRNA-129-5p)	[235–245]
ATB	Up	Bladder cancer; Prostate carcinoma	Cell proliferation, migration and invasion; mitogenic; epithelial-mesenchymal transition (microRNA-126, KRAS,)	[246, 247]
BC087858	Up	Non-small-cell lung cancer	Cells invasion; resistance to EGFR-TKIs (ZEB1, Snail.)	[248]
Linc00659	Up	Colorectal cancer	Cell growth inhibition and apoptosis	[249]
Linc00152	Up	Lung cancer; Gallbladder cancer	Cell proliferation, invasion, migration, apoptosis, and G1 phase rates	[250, 251]
Linc00462	Up	Hepatocellular carcinoma	Cell proliferation, invasion and migration	[252]
Linc01296	Up	Prostate cancer; Colorectal cancer	Tumorigensis, cell proliferation, migration, invasion, and liver metastasis; epithelial-mesenchymal transition; chemoresistance to 5-fluorouracil (miRNA-26a, mucin1, GALNT3)	[253, 254]
Linc003121	Down	Thyroid cancer	Cell proliferation, Invasion, and tumorigenicity	[255]
UCA1	Up	Gastric cancer; Bladder cancer	Cell proliferation, migration, invasion, apoptosis and cell cycle	[256–259]
ecCEBPA	Up	Gastric cancer; Hepatic cancer	Disease progression	[257, 260]
Ftx	Up	Hepatocellular carcinoma	Cell growth (miRNA-545, RIG-I)	[261]
RMEL3	Up	Melanoma	Cell survival and proliferation (PTEN)	[262]
LncARSR	Up	Hepatocellular Carcinoma	Doxorubicin resistance (PTEN)	[206]
BDLNR	Up	Cervical cancer	Cell proliferation, migration, and death; anti-cancer effects of baicalein (YBX1, PIK3CA promoter)	[263]
ANRIL	Up	Cervical cancer; Osteosarcoma; Gliomas	Cell proliferation, migration, invasion, and apoptosis (miRNA-34a, Sirt1)	[264–266]
ROR	Up	Non-small-cell lung cancer	Cell proliferation, migration, and invasion; cisplatin resistance	[267]
PlncRNA-1	Up	Colorectal cancer	Cell proliferation, migration, invasion, and apoptosis	[268]
MYD88	Up	Hepatocellular carcinoma;	Cell proliferation and metastasis (H3K27Ac)	[269]
RP4	Down	Colorectal cancer	Cell proliferation, growth, and early apoptosis (SH3GLB1, miRNA-7-5p)	[270]
OIP5-AS1	Down	Osteosarcoma, myeloma	Cell growth; cisplatin resistance (miRNA-340-5p, LPAATbeta, miRNA-410, KLF10)	[201, 213]
MEG3	Down	Endometrial carcinoma; Breast cancer; Cervical cancer; Pancreatic cancer; Lymphoma; Gliomas	Cell proliferation, migration, invasion, metastasis, and apoptosis; autophagy; glycolysis; epithelial-mesenchymal transition; chemoresistance (Combine directly with PI3K, miRNA-21, cytomembrane translocation of AKT)	[271–277]
GAS5	Down	Colorectal cancer; Esophageal squamous cell carcinoma; Breast cancer; Malignant pleural mesothelioma; Osteosarcoma; Prostate cancer	Cell proliferation and migration, viability, migration and invasion; apoptotic responses to conventional chemotherapies (miRNA-203a, TIMP2, miRNA-196a-5p, FOXO1)	[66–72]
RNA-422	Up	Colorectal cancer	Cell proliferation, migration, and invasion	[278]

## PI3K inhibitors

PI3K are believed to be one of the key therapeutic targets for cancer treatment based on the observation that hyperactivity of PI3K signaling is significantly correlated with human tumor progression, increased tumor microvessel density and enhanced chemotaxis and invasive potential of cancer cells. Enormous efforts have been dedicated to the development of drugs targeting PI3K signaling, many of which are currently employed in clinical trials evaluation. Important ongoing clinical trials with PI3K-targeted therapies were summarized in Table 2. PI3K inhibitors are subdivided into dual PI3K/mTOR inhibitors, pan-PI3K inhibitors and isoform-specific inhibitors. The drugs targeting PI3K in clinical trial were shown in Table 3 and Fig. 2.

**Table 2:** Important ongoing clinical trials with PI3K-targeted therapies

Conditions	Sample size	Design	Phase	Status	Trial number
NVP-BEZ235 (BEZ235, Dactolisib) Dual PI3K/mTOR inhibitor					
Acute Lymphoblastic Leukemia; Acute Chronic Myelogenous Leukemia With Crisis of Blast Cells	23	BEZ235	I	Active not recruiting	NCT01756118
GDC-0084 (RG7666) Dual PI3K/mTOR inhibitor					
Glioblastoma, Adult	66	GDC-0084	II	Recruiting	NCT03522298
Brain and Central Nervous System Tumors	41	Radiation therapy+ GDC-0084	I	Not yet recruiting	NCT03696355
GDC-0980 (Apitolisib, RG7422) Dual PI3K/mTOR inhibitor					
Prostate Cancer	273	Abiraterone Acetate +/− (GDC-0980/Ipatasertib)	I/II	Active not recruiting	NCT01485861
LY3023414 Dual PI3K/mTOR inhibitor					
Endometrial Cancer; Recurrent Endometrial Cancer	25	LY3023414	II	Recruiting	NCT02549989
Advanced Malignant Solid Neoplasm; Ann Arbor Stage III/IV Childhood Non-Hodgkin Lymphoma	–	LY3023414	II	Recruiting	NCT03155620
Metastatic Colorectal Neoplasm; Metastatic Breast Cancer	205	Prexasertib+Cisplatin/Cetuximab/Pemetrexed/5-FU/LY3023414	I	Recruiting	NCT02124148
Advanced or Metastatic Solid Tumors	163	LY3039478 + LY3023414/Taladegib/Abemaciclib/Cisplatin/Gemcitabine/Carboplatin	I	Recruiting	NCT02784795
NSCLC	150	Abemaciclib+LY3023414/Pemetrexed/Gemcitabine/Ramucirumab/Pembrolizumab	I	Active not recruiting	NCT02079636
Prostate Cancer Metastatic	144	Enzalutamide +/− LY3023414	II	Recruiting	NCT02407054
Advanced Non-Hodgkin Lymphoma; Metastatic Breast Cancer; Advanced Mesothelioma; Advanced NSCLC	130	LY3023414 + Midazolam/Fulvestrant OR LY3023414 + Pemetrexed/Cisplatin OR LY3023414 +/− (Abemaciclib+ Letrozole)	I	Recruiting	NCT01655225
Pancreatic Ductal Adenocarcinoma	231	Abemaciclib+/− LY3023414 VS Gemcitabine/Capecitabine	II	Active not recruiting	NCT02981342
Breast Neoplasms	198	LY3023414 + LY2835219 + Fulvestrant	I	Recruiting	NCT02057133
Advanced Malignant Solid Neoplasm; Ann Arbor Stage III/ IV Non-Hodgkin Lymphoma	144	LY3023414	II	Recruiting	NCT03213678
Endometrial Cancer	62	(LY3023414 + Abemaciclib) +/− Letrozole	II	Not yet recruiting	NCT03675893
PF-05212384 (Gedatolisib, PKI-587) Dual PI3K/mTOR inhibitor					
Therapy-related Acute Myeloid Leukemia and Myelodysplastic Syndrome; Relapsed Acute Myeloid Leukemia; de Novo Acute Myeloid Leukemia at Diagnostic	10	PF-05212384	II	Active not recruiting	NCT02438761
Neoplasm	124	PF-05212384 + Docetaxel/Cisplatin/Dacomitinib	I	Recruiting	NCT01920061
Lung Cancer Squamous Cell; Solid Tumors; Head & Neck Cancer; Pancreatic Cancer	96	PF-05212384 + Palbociclib	I	Recruiting	NCT03065062
NSCLC	51	PF-05212384/Paclitaxel/Carboplatin	I/II	Recruiting	NCT02920450
Breast Cancer; NSCLC; Ovary Cancer; Endometrial Cancer; SCLC	40	PF-05212384 + Paclitaxel+Carboplatin	I	Recruiting	NCT02069158
ER+/HER2- Breast Cancer	18	PF-05212384 + Fulvestrant+ Palbociclib	I	Recruiting	NCT02626507
Breast Cancer	80	Hydrpxychloroquine+/− PF-05212384	I/II	Not yet recruiting	NCT03400254
Breast Cancer	120	PF-05212384 + Palbociclib+/−Letrozole/Fulvestrant	I	Recruiting	NCT02684032
Triple Negative Breast Cancer; Metastatic Breast Cancer	18	PF-05212384 + PTK7-ADC	I	Recruiting	NCT03243331
PQR309 (Bimiralisib) Dual PI3K/mTOR inhibitor					
Lymphoma	72	PQR309	I/II	Recruiting	NCT02249429
Lymphoma; Non-Hodgkin Lymphoma	72	PQR309	II	Recruiting	NCT03127020
Primary Central Nervous System Lymphoma	21	PQR309	II	Not yet recruiting	NCT03120000
Metastatic Breast Cancer	60	PQR309 + Eribulin	I/II	Recruiting	NCT02723877
P7170 Dual PI3K/mTOR inhibitor					
Advanced Refractory Solid Tumors	60	P7170	I	Suspended	NCT01762410
SF-1126 Dual PI3K/mTOR inhibitor					
Advanced Hepatocellular Carcinoma	14	SF-1126	I	Recruiting	NCT03059147
Advanced Castrate-resistant Prostate Cancer; Squamous NSCLC; Triple Negative Breast Cancer	180	AZD8186+/−Abiraterone Acetate/AZD2014	I	Recruiting	NCT01884285
Copanlisib (BAY 80–6946) PI3Kδ/α inhibitor					
Recurrent Endometrial, Ovarian, Primary Peritoneal, or Fallopian Tube Cancer	44	Copanlisib+Niraparib	I	Not yet recruiting	NCT03586661
Head and Neck Squamous Cell Carcinomas	32	Copanlisib+Cetuximab	I/II	Recruiting	NCT02822482
Endometrial cancer	84	Copanlisib	II	Suspended	NCT02728258
HR+, HER2-, Stage I-IV Breast Cancer	102	Copanlisib+Letrozole+/-Palbociclib	I/II	Recruiting	NCT03128619
HER2+ Breast Cancer	19	Copanlisib +Trastuzumab	I	Recruiting	NCT02705859
Non-Hodgkin Lymphoma	25	Copanlisib	I/II	Active not recruiting	NCT02342665
Mature T-Cell and NK-Cell Neoplasm	36	Copanlisib+Gemcitabine	I/II	Recruiting	NCT03052933
Advanced or Metastatic Solid Tumor	65	Copanlisib+Rogaratinib	I	Recruiting	NCT03517956
Medical Oncology	51	Copanlisib+/-Itraconazole/ Rifampin	I	Active not recruiting	NCT02253420
Mixed Tumor, Malignant	130	Copanlisib	I/II	Recruiting	NCT03458728
Biliary Carcinoma; Gall Bladder Carcinoma; Cholangiocarcinoma; Gastrointestinal Tumor	25	Copanlisib+Gemcitabine+Cisplatin	II	Recruiting	NCT02631590
Refractory/Recurrent Primary Central Nervous System Lymphoma	45	Copanlisib+Ibrutinib	I/II	Not yet recruiting	NCT03581942
Marginal Zone Lymphoma	56	Copanlisib+Rituximab	II	Not yet recruiting	NCT03474744
Large B-Cell Lymphoma	99	Copanlisib+Nivolumab	II	Not yet recruiting	NCT03484819
Ann Arbor Stage III/IV Lymphoma; Metastatic Malignant; Solid Neoplasm	50	Copanlisib+Nivolumab	I	Recruiting	NCT03502733
Non-Hodgkin Lymphoma	450	Rituximab+Copanlisib/Placebo	III	Recruiting	NCT02367040
Non-Hodgkin Lymphoma	227	Copanlisib	II	Active not recruiting	NCT01660451
Non-Hodgkin Lymphoma	25	Copanlisib	III	Active not recruiting	NCT02369016
Non-Hodgkin Lymphoma	12	Copanlisib	I	Recruiting	NCT03498430
Non-Hodgkin Lymphoma	546	Standard Immunochemotherapy+/− Copanlisib	III	Recruiting	NCT02626455
Buparlisib (BKM120 NVP-BKM120) Class I PI3K inhibitor					
Metastatic Transitional Cell Carcinoma of the Urothelium	35	Buparlisib	II	Active not recruiting	NCT01551030
Metastatic Squamous Neck Cancer With Occult Primary Squamous Cell Carcinoma;	30	Buparlisib+Cetuximab	I/II	Active not recruiting	NCT01816984
Head and Neck Cancer	170	Buparlisib	II	Recruiting	NCT01737450
NSCLC	37	Buparlisib+Erlotinib	II	Active not recruiting	NCT01487265
NSCLC	38	Buparlisib+Gefitinib		Active not recruiting	NCT01570296
Advanced Squamous Cell Cancer of Head and Neck	23	Radiotherapy+Buparlisib+ Cisplatin	I	Active not recruiting	NCT02113878
Breast Cancer	106	Buparlisib+lapatinib	I/II	Suspended (Data analysis)	NCT01589861
Breast Cancer	1149	Buparlisib/Placebo+Fulvestrant	III	Active not recruiting	NCT01610284
Breast Cancer	110	Buparlisib	II	Active not recruiting	NCT01790932
Metastatic Breast Cancer	47	Buparlisib+Capecitabine+/− (Trastuzumab/Lapatinib) OR BYL719+ Capecitabine	I	Active not recruiting	NCT01300962
Breast Cancer Patients With Brain Metastases	10	Buparlisib/Capecitabine	II	Active not recruiting	NCT02000882
Pre-menopausal Breast Cancer	40	Buparlisib/BYL719 + Tamoxifen+Goserelin Acetate	I	Active not recruiting	NCT02058381
Ovarian Cancer; Breast Cancer	118	Buparlisib/BYL719+ Olaparib	I	Active not recruiting	NCT01623349
Glioblastoma Multiforme	88	Buparlisib+Bevacizumab	I/II	Active not recruiting	NCT01349660
Glioblastoma	65	Buparlisib+/-Surgery	II	Active not recruiting	NCT01339052
Thyroid Cancers	47	Buparlisib	II	Active not recruiting	NCT01830504
Thymoma	14	Buparlisib	II	Active not recruiting	NCT02220855
Malignant Melanoma; Metastases	22	Buparlisib	II	Recruiting	NCT02452294
Melanoma	140	LGX818 + MEK162+/−(Buparlisib/LEE011/ BGJ398/ INC280)	II	Active not recruiting	NCT02159066
Metastatic Colorectal Cancer	22	Buparlisib+Panitumumab	I/II	Active not recruiting	NCT01591421
Relapsed or Refractory Indolent B-Cell Lymphoma	18	Buparlisib+Rituximab	I	Active not recruiting	NCT02049541
Chronic Lymphocytic Leukemia	14	Buparlisib	II	Active not recruiting	NCT02340780
Recurrent/ Refractory Chronic Lymphocytic Leukemia; Recurrent/ Refractory Small Lymphocytic Lymphoma	1	Buparlisib+Ofatumumab/Ibrutinib	I	Active not recruiting	NCT02614508
Mantle Cell Lymphoma; Follicular Lymphoma; Diffuse Large B Cell Lymphoma	37	Buparlisib+Ibrutinib	I	Active not recruiting	NCT02756247
Duvelisib (IPI-145) PI3Kδ/γ inhibitor					
Indolent Non-Hodgkin Lymphoma	129	Duvelisib	II	Active not recruiting	NCT01882803
Relapsed/Refractory T-cell Lymphomas	88	Duvelisib+Romidepsin/ Bortezomib	I	Recruiting	NCT02783625
Peripheral T-cell Lymphoma	120	Duvelisib	II	Recruiting	NCT03372057
Chronic Lymphocytic Leukemia	47	Duvelisib+Venetoclax	I/II	Recruiting	NCT03534323
Hematologic Malignancy	500	Duvelisib	II	Active not recruiting	NCT02711852
Chronic Lymphocytic Leukemia; Small Lymphocytic Lymphoma	150	Duvelisib VS Ofatumumab	III	• Enrolling by invitation	NCT02049515
Chronic Lymphocytic Leukemia; Small Lymphocytic Lymphoma	300	Duvelisib VS Ofatumumab	III	Active not recruiting	NCT02004522
Chronic Lymphocytic	50	Duvelisib	II	Recruiting	NCT03370185
Leukemia; Small Lymphocytic Lymphoma					
Chronic Lymphocytic Leukemia	32	Duvelisib+Fludarabine+Cyclophosphamide+Rituximab	I/II	Active not recruiting	NCT02158091
RP6530 (Tenalisib) PI3Kδ/γ inhibitor					
Peripheral T-Cell Lymphoma; Cutaneous T-Cell Lymphoma	58	RP6530	I	Active not recruiting	NCT02567656
Classical Hodgkin Lymphoma	57	RP6530 + Pembrolizumab	I	Recruiting	NCT03471351
Taselisib (GDC-0032) PI3Kα/β/γ inhibitor					
Recurrent/ Stage IV Squamous Cell Lung Carcinoma	59	Taselisib	II	Active not recruiting	NCT02785913
Metastatic Breast Cancer; Recurrent Breast Cancer	76	Taselisib+Trastuzumab emtansine +/− Pertuzumab OR Pertuzumab+Trastuzumab+/− Paclitaxel	I	Recruiting	NCT02390427
Androgen Receptor Positive Triple Negative Metastatic Breast Cancer	73	Taselisib+Enzalutamide	I/II	Active not recruiting	NCT02457910
Breast Cancer	290	Tamoxifen+ Taselisib/Placebo	I/II	Recruiting	NCT02285179
Breast Cancer	631	Fulvestrant+ Taselisib/Placebo	III	Active not recruiting	NCT02340221
PIK3CA-Related Overgrowth	30	Taselisib	I/II	Recruiting	NCT03290092
Solid Cancers; Non-Hodgkin Lymphoma	724	Taselisib+/-Fulvestrant/Letrozole/Midazolam/ Fulvestrant	I	Active not recruiting	NCT01296555
Advanced Refractory Solid Tumors; Lymphomas; Multiple Myeloma	6452	Molecular Analysis for Therapy Choice Screening Trial	II	Recruiting	NCT02465060
KA2237 PI3Kβ/γ inhibitor					
B Cell Lymphoma	53	KA2237	I	Recruiting	NCT02679196
BYL719 (Alpelisib) PI3Kα inhibitor					
PIK3CA Mutated Advanced Breast Cancer	90	BYL719 VS Chemotherapy	II	Recruiting	NCT03386162
Breast Cancer	23	BYL719 + LJM716+ Trastuzumab	I	Active not recruiting	NCT02167854
Breast Cancer	44	BYL719 + Nab-Paclitaxel	I/II	Active not recruiting	NCT02379247
HER2+ Metastatic Breast Cancer	17	BYL719 + Ado-Trastuzumab Emtansine	I	Active not recruiting	NCT02038010
Metastatic Breast Cancer	34	BYL719	II	Recruiting	NCT02506556
Malignant Neoplasm of Breast	28	BYL719 + Enzalutamide	I	Not yet recruiting	NCT03207529
Pancreatic Cancer	15	BYL719 + Gemcitabine+(Nab)-Paclitaxel	I	Active not recruiting	NCT02155088
Breast Cancer	572	Fulvestrant+ BYL719/Placebo	III	Active not recruiting	NCT02437318
Premenopausal Patients With HR+, HER2- Locally Advanced or Metastatic Breast Cancer	40	BYL719/BKM120 + Tamoxifen+Goserelin Acetate	I	Active not recruiting	NCT02058381
Advanced or Metastatic ER+ Breast Cancer	312	LSZ102+/− LEE011/BYL719	I	Recruiting	NCT02734615
Metastatic or Locally-advanced Unresectable Breast Cancer	52	BYL719 + Letrozole/Exemestane	I	Active not recruiting	NCT01870505
Breast Cancer	160	BYL-719 + Fulvestrant/Letrozole	II	Recruiting	NCT03056755
ER+ Breast Cancer; HER2-negative Breast Cancer; Invasive Ductal Breast Carcinoma	46	BYL719 + Letrozole	I	Active not recruiting	NCT01791478
Breast Cancer	253	Letrozole+BYL719/LEE011/ Both	I	Recruiting	NCT01872260
Metastatic Breast Cancer	47	BMK120 + Capecitabine+/− Trastuzumab/Lapatinib OR BYL719+ Capecitabine	I	Active not recruiting	NCT01300962
Head and Neck Cancer and Esophageal Cancer Patient	259	BYL719/Poziotinib/Nintedanib/Abemaciclib/(Durvalumab+Tremelimumab)	II	Recruiting	NCT03292250
Head and Neck Squamous Cell Cancer	30	BYL719	N/A	Recruiting	NCT03138070
Recurrent or Metastatic Squamous Cell Carcinoma of Head and Neck	43	BYL719	II	Recruiting	NCT02145312
Head and Neck Squamous Cell Cancer	16	BYL719 + Cetuximab+IMRT (Intensity-Modulated Radiation Therapy)	I	Active not recruiting	NCT02282371
Locoregionally Advanced Squamous Cell Carcinoma of Head and Neck	36	BYL719 + Cisplatin+Radiation (Intensity modulated radiation therapy)	I	Recruiting	NCT02537223
Uveal Melanoma	30	BYL719 + AEB071	I	Active not recruiting	NCT02273219
Rectal Cancer	24	BYL719 + Capecitabine+Radiation	I	Recruiting	NCT02550743
Colorectal Cancer	150	LGX818 + Cetuximab+/− BYL719	I/II	Active not recruiting	NCT01719380
Patients With Gastrointestinal Stromal Tumor	56	BYL719 + ST571	I	Active not recruiting	NCT01735968
Adenocarcinoma Lung Cancer; Squamous Cell Lung Carcinoma	67	BYL719/AUY922/INC280/LDK378/MEK162	II	Active not recruiting	NCT02276027
CDKN2A-p16+; Human Papillomavirus+ Oropharyngeal Squamous Cell Carcinoma	14	BYL719 + Surgery	II	Not yet recruiting	NCT03601507
Breast Neoplasms; Kidney Neoplasms; Pancreatic Neuroendocine Neoplasms	79	BYL719 + Everolimus/Exemestane/Both	I	Active not recruiting	NCT02077933
Advanced Solid Tumors With an Alteration of the PIK3CA Gene; ER+ Breast Cancer	221	BYL719+/-Fulvestrant	I	Active not recruiting	NCT01219699
Solid Tumors	41	BYL719 + Cisplatin	I	Recruiting	NCT02620839
Ovarian Cancer; Breast Cancer	118	Olaparib+BYL719/BKM120	I	Active not recruiting	NCT01623349
Meningioma	25	BYL719 + Trametinib	I	Not yet recruiting	NCT03631953
CAL-101 (GS-1101, Idelalisib) PI3Kδ inhibitor					
Metastasis/Recurrence NSCLC	40	CAL-101 + Pembrolizumab	I/II	Recruiting	NCT03257722
Waldenstrom Macroglobulinemia	50	Obinutuzumab	II	Active not recruiting	NCT02962401
Chronic Lymphocytic Leucemia	62	CAL-101 + Bendamustine+GA101	II	Recruiting	NCT02445131
Chronic Lymphocytic LeukemiaSmall Lymphocytic Lymphoma	50	CAL-101 + Ofatumumab	II	Suspended	NCT02135133
Follicular Non-Hodgkin Lymphoma Refractory	260	CAL-101	N/A	Recruiting	NCT03568929
Chronic Lymphocytic Leukemia	42	CAL-101 + Rituximab+Venetoclax	I	Not yet recruiting	NCT03639324
Chronic Lymphocytic Leukemia	104	CAL-101 + Rituximab	N/A	Not yet recruiting	NCT03545035
Diffuse Large B-Cell	36	CAL-101 + (Rituximab+Ifosfa	I	Recruiting	NCT03349346
Lymphoma; Mediastinal B-cell Lymphoma		mide+Carboplatin+Etoposide) (RICE)			
Chronic Lymphocytic Leukemia	35	CAL-101 + Tirabrutinib+/− Obinutuzumab	II	Recruiting	NCT02968563
Chronic Lymphocytic Leukemia; Small Lymphocytic Lymphoma	24	MOR00208 + CAL-101/ Venetoclax	II	Recruiting	NCT02639910
Chronic Lymphocytic Leukemia	308	Acalabrutinib VS Rituximab + CAL-101/Bendamustine	III	Recruiting	NCT02970318
Recurrent Chronic Lymphocytic Leukemia; Extranodal Marginal Zone Lymphoma; Follicular Lymphoma	68	Pembrolizumab+/-CAL-101/Ibrutinib	II	Recruiting	NCT02332980
B-cell Malignancies	197	Tirabrutinib+/-CAL-101/Entospletinib+/− Obinutuzumab	I	Active not recruiting	NCT02457598
Chronic Lymphocytic Leukemia; Peripheral T-cell Lymphoma	123	TRU-016 + Rituximab/ Obinutuzumab/Ibrutinib/ Bendamustine OR TRU-016 + Rituximab+CAL-101	I	Recruiting	NCT01644253
Acute Lymphoblastic Leukemia; Acute Myeloid Leukemia	24	Personalized Kinase Inhibitor Therapy Combined With Chemotherapy	I	Recruiting	NCT02779283
Non-Hodgkin Lymphoma	30	CAL-101	N/A	Recruiting	NCT02928510
Hematological Malignancies	150	CAL-101 VS Ibrutinib (Side Effects)	N/A	Recruiting	NCT02824159
Recurrent Chronic Lymphoid Leukemia	3	ACY-1215+ CAL-101/Ibrutinib	I	Active not recruiting	NCT02787369
Chronic Lymphocytic Leukemia	416	Rituximab+Bendamustine+ Placebo/ CAL-101	III	Active not recruiting	NCT01569295
Follicular Lymphoma	240	CAL-101	III	Recruiting	NCT02536300
B Cells-Tumors; B Cell Chronic Lymphocytic Leukemia; Follicular Lymphoma; Mantle Cell Lymphoma; Large B-Cell Diffuse Lymphoma	60	CAL-101 VS Placebo	I	Recruiting	NCT03151057
Chronic Lymphocytic Leukemia; Small Lymphocytic Lymphoma	24	MOR00208 + CAL-101/ Venetoclax	II	Active not recruiting	NCT02639910
Diffuse Large B Cell Lymphoma	72	CAL-101	II	Recruiting	NCT03576443
B-Cell Non-Hodgkin Lymphoma	34	CAL-101	II	Recruiting	NCT03133221
Chronic Lymphocytic Leukemia	20	CAL-101 + Rituximab	N/A	Recruiting	NCT02993536
Chronic Lymphocytic Leukaemia	150	CAL-101 + Rituximab	N/A	Not yet recruiting	NCT03582098
GSK2636771 PI3Kβ inhibitor					
Gastric Cancer	400	Biomarker Screening	N/A	Recruiting	NCT02951091
Advanced Gastric Adenocarcinoma	66	GSK2636771+ Paclitaxel	I/II	Recruiting	NCT02615730
Metastatic Castration-Resistant Prostate Cancer	64	GSK2636771+ Enzalutamide	I	Recruiting	NCT02215096
Melanoma and Other Malignant Neoplasms of Skin; Metastatic Melanoma	41	GSK2636771 + Pembrolizumab	I/II	Recruiting	NCT03131908
Advanced Malignant Solid Neoplasm	–	Patients with PTEN mutation, deletion, expression or loss were given GSK2636771	II	Recruiting	NCT02465060
INCB050465 (Parsaclisib) PI3Kδ inhibitor					
MPN (Myeloproliferative Neoplasms)	78	INCB050465 + Ruxolitinib	II	Recruiting	NCT02718300
Advanced Solid Tumors	237	Pembrolizumab+Itacitinib/ INCB050465	I	Recruiting	NCT02646748
Advanced Solid Tumors	159	Itacitinib+Epacadostat/ INCB050465	I	Active, not recruiting	NCT02559492
Solid Tumors; Advanced Malignancies; Metastatic Cancer	80	Ia:INCB052793 Ib:INCB052793 + (Gemcitabine+Nab-Paclitaxel+Dexamethasone+Carfilzomib/+Bortezomib+Lenalidomide+Azacitidine+INCB052793 + Pomalidomide+INCB050465) II:INCB052793 + Azacitidine+ INCB039110	I/II	Active not recruiting	NCT02265510
Unresectable or Metastatic Solid Tumors	100	INCMGA00012 + Epacadostat / INCB050465	I	Recruiting	NCT03589651
Primary Sjögren’s Syndrome	12	INCB050465	II	Not yet recruiting	NCT03627065
Lymphoma	120	INCB050465	II	Recruiting	NCT03235544
Lymphoma	120	INCB050465+/-CITADEL-204	II	Recruiting	NCT03144674
Lymphoma	60	INCB050465	II	Active not recruiting	NCT02998476
Lymphoma	18	INCB050465	I	Recruiting	NCT03314922
Lymphoma	45	INCB050465 + Bendamustine +Obinutuzumab	I	Recruiting	NCT03039114
Lymphoma	100	INCB050465	II	Recruiting	NCT03126019
B-Cell Malignancies	88	INCB050465+/-Itacitinib OR INCB050465 + Rituximab+Ifosfamide+Carboplatin+Etoposide	I/II	Active not recruiting	NCT02018861
Relapsed/ Refractory Diffuse Large B-Cell Lymphoma	25	INCB050465 + INCB053914	I	Not yet recruiting	NCT03688152
B-cell Lymphoma	81	INCB050465 + Rituximab+/− Bendamustine OR INCB050465+ Ibrutinib	I	Recruiting	NCT03424122
Serabelisib (INK-1117,MLN-1117,TAK-117) PI3Kα inhibitor					
Advanced Solid Tumor	30	Serabelisib+TAK-228+ Paclitaxel	I	Not yet recruiting	NCT03154294
Clear-cell Metastatic Renal Cell Carcinoma	96	MLN0128+/-Serabelisib VS Everolimus	II	Active not recruiting	NCT02724020
Endometrial Neoplasms	242	Paclitaxel+/− MLN0128 OR MLN0128+/− Serabelisib	II	Recruiting	NCT02725268
Triple Negative Breast Cancer	20	TAK-228 + Serabelisib+ Cisplatin+Nab Paclitaxel	II	Recruiting	NCT03193853
ME401 (PWT-143) PI3Kδ inhibitor					
Chronic Lymphocytic Leukemia (CLL) Small Lymphocytic Lymphoma (SLL), B-cell Non-Hodgkin Lymphoma	133	ME401+/−Rituximab	I	Recruiting	NCT02914938
Umbralisib (RP5264, TGR-1202) PI3Kδ inhibitor					
Marginal Zone Lymphoma; Waldenstrom Macroglobulinemia	30	Umbralisib	II	Recruiting	NCT03364231
Chronic Lymphocytic Leukemia	30	Ublituximab +Umbralisib + Venetoclax	I/II	Recruiting	NCT03379051
Follicular Lymphoma	150	Obinutuzumab+ Umbralisib / lenalidomide/Chemotherapy	II	Recruiting	NCT03269669
Non-Hodgkin Lymphoma; Chronic Lymphocytic Leukemia	50	TG-1701 +/− (Ublituximab + Umbralisib)	I	Recruiting	NCT03671590
Chronic Lymphocytic Leukemia; B-cell Non-Hodgkin Lymphoma	36	Umbralisib +Pembrolizumab	I	Recruiting	NCT03283137
Chronic Lymphocytic Leukemia/Small Lymphocytic Lymphoma; Mantle Cell Lymphoma	45	Umbralisib+Ibrutinib	I	Active not recruiting	NCT02268851
CUDC-907 (Fimepinostat) PI3Kα/β/δ and HDAC1/2/3/10 inhibitor					
Advanced/Relapsed Solid Tumors	60	CUDC-907	I	Recruiting	NCT02307240
Lymphoma; Neuroblastoma; Brain Tumor; Solid Tumor	44	CUDC-907	I	Recruiting	NCT02909777
Multiple Myeloma; Lymphoma	88	CUDC-907	I	Active not recruiting	NCT01742988
Relapsed and/or Refractory Diffuse Large B-cell Lymphoma Including With Myc Alterations	200	CUDC-907	II	Recruiting	NCT02674750
Rigosertib (ON-01910) PI3K and PIk-1 inhibitor					
Leukemia; Myelofibrosis; Anemia; Splenomegaly	35	Rigosertib	II	Recruiting	NCT02730884
Myelodysplastic Syndromes	36	Rigosertib	I	Suspended	NCT02075034
Myelodysplastic Syndromes	45	Rigosertib	II	Active not recruiting	NCT01904682
Myelodysplastic Syndromes; MDS; RAEB; Chronic Myelomonocytic Leukemia	299	Rigosertib	III	Active not recruiting	NCT01241500
Myelodysplastic Syndromes; Refractory Anemia With Excess Blasts; Chronic Myelomonocytic Leukemia; Cytopenia	67	Rigosertib	III	Active not recruiting	NCT01928537
Myelodysplastic Syndromes	12	Rigosertib	I	Recruiting	NCT03495167
Myelodysplastic Syndrome; Acute Myeloid Leukemia; Chronic Myelomonocytic Leukemia	45	Rigosertib+Azacitidine	I/II	Active not recruiting	NCT01926587
Myelodysplastic Syndrome; MDS; Refractory Anemia With Excess Blasts; RAEB	360	Rigosertib VS. Any approved or standard-of-care therapy	III	Recruiting	NCT02562443

Abbreviations: *NSCLC* Non-small cell lung cancer, *SCLC* Small cell lung cancer, *ER* Estrogen Receptor, *PR* Progesterone receptor

**Table 3:** Drugs targeting PI3K in clinical trial

Compound	Terminated	Phase I	Phase II	Phase III	FDA approved
Dual PI3K/mTOR inhibitor	BGT-226 (Novartis) DS-7423 (Daiichi Sankyo) PF-04691502 (Pfizer) PKI-179 (Pfizer)	GSK458/Omipalisib(GlaxoSmithKline) P7170 (Piramal) SB2343/VS-5584 (Verastem)	BEZ235/Dactolisib (Novartis) GDC-0084 (Novogen) GDC-0980/Apitolisib (Genentech) LY3023414 (Eli Lilly) PQR309/Bimiralisib (PIQUR Therapeutics) XL765/Voxtalisib (Sanofi) SF-1126 (SignalRx)	PF-05212384/gedatolisib/ PKI-587 (Pfizer)	
Pan-PI3K inhibitor	GDC-0941/Pictilisib (Genentech) PX-866 (Oncothyreon) TG100–115 (Sanofi)	CH5132799 (TohokuNiproPharm)	XL147/ Pilaralisib (Sanofi) ZSTK474 (Zenyaku Kogyo)	BKM-120/Buparlisib (Novartis)	BAY80–6946/ Copanlisib (Bayer)
Isoform-specific PI3K inhibitor	AZD8835 (AstraZeneca) δ/α WX-037 (Wilex) α	AZD8186 (AstraZeneca) β/δ KA2237 (Karus Therapeutics) β/δ GS-9820/CAL-120 (Gilead) β/δ ME401/PWT-143 (MEI Pharma) δ	AMG 319 (Amgen) δ GSK2636771 (GlaxoSmithKline) β INCB050465/Parsaclisib (Incyte) δ Serabelisib/INK-1117 (Takeda) α Umbralisib/TGR-1202 (TG Therapeutics) δ RP6530/Tenalisib(Rhizen Pharmaceuticals) δ/γ	GDC-0032/Taselisib (Genentech) α/δ/γ BYL719/Alpelisib (Novartis) α	Duvelisib/IPI-145 (Infinity) δ/γ CAL-101/idelalisib (Gilead) δ
Others			CUDC-907/Fimepinostat (Curis)	Rigosertib/ON-01910 (Onconova Therapeutics)

**Fig. 2:** Targeting PI3K/Akt/mTOR pathway in cancer

### Dual PI3K/mTOR inhibitors

#### NVP-BEZ235 (Dactolisib)

NVP BEZ235 (dactolisib) is a dual PI3K/mTOR inhibitor and is currently in Phase I/II clinical trials. It is an imidazo [4,5-c] quinoline derivative compound that binds to the ATP-binding cleft of PI3K and mTOR kinase, inhibiting their catalytic activities [25]. BEZ235 exhibited satisfactory anticancer effects in preclinical studies in several types of cancer, including the following: triple-negative breast cancer, lung cancer, melanoma, colorectal cancer, renal cancer, prostate cancer, lymphoma, and mucinous adenocarcinoma of the ovary [73–85]. However, the clinical trials of BEZ235 were not satisfactory. A phase I study investigated maximum tolerated dose (MTD), recommended dose for expansion (RDE), safety and antitumor activity of BEZ235, in combination with abiraterone acetate [86]. In this study, dose escalation was stopped after 200 mg bid due to challenging safety and tolerability profile; the most common adverse events (AEs) were diarrhea (78%), nausea (61%) and stomatitis (39%). Moreover, no objective response and few prostate specific antigen (PSA) decreases were reported. Limited efficacy and poor tolerance of BEZ235 combined with everolimus (BEZ235: 200, 400, or 800 mg daily; everolimus: 2.5 mg daily; 28-day cycles) in patients with advanced solid malignancies were reported in a phase Ib trial [87].

In a Phase II Study, BEZ235 was poorly tolerated by patients with everolimus-resistant pancreatic neuroendocrine tumor at 400 or 300 mg bid doses, and the estimated 16-week progression-free survival (PFS) rate was 51.6% [88]. Treatment-related grade 3/4 AEs including hyperglycaemia, nausea, diarrhoea, and vomiting occurred in 72.7% patients at 400 mg and 40.0% patients at 300 mg; 95.0% of the patients in the 300 mg group and all patients in the 400 mg group experienced at least one AE relating to the treatment [88]. Treatment with BEZ235 in mTOR inhibitor-naive patients with advanced pancreatic neuroendocrine tumors demonstrated poorer efficacy and tolerability compared with everolimus in another Phase II study [89]. Phase I studies of BEZ235 in patients with advanced breast cancer and advanced renal cancer, reported that BEZ235 was not enough to achieve a satisfactory antitumor effect with a favorable safety profile. Currently, several clinical studies of BEZ235 among patients with relapsed or refractory acute leukemia and patients with metastatic breast cancer are ongoing.

#### GDC-0980 (Apitolisib, RG7422)

GDC-0980 (apitolisib, RG7422) is a potent, orally bioavailable inhibitor of class I PI3K and mTOR kinase (TORC1/2). Several preclinical studies have assessed this agent’s activity in a variety of solid tumors. A phase I trial assessed the safety, tolerability, and preliminary antitumor effects of GDC-0980 in patients with solid tumors [90]. In this study, 2–70 mg daily GDC-0980 was administered to patients for days 1–21 or 1–28 of 28-day cycles. The main AEs from this agent were hyperglycemia, rash, liver dysfunction and diarrhea. This phase I study concluded that GDC-0980 has a narrow therapeutic window, and dose of 40 mg 28/28 days was reasonably tolerated. More recently, a single arm, open-label trial phase II study in recurrent or persistent endometrial carcinoma patients reported that anti-tumor activity of 40 mg GDC-0980 daily was limited by tolerability, especially in diabetic patients, and patients with mutations of PI3K pathway may benefit more from GDC-0980 [91].

In another phase II study, 85 patients with metastatic renal cell carcinoma were randomly assigned to apitolisib 40 mg QD or to everolimus 10 mg QD. Patients receiving GDC-0980 were shown to have poorer median PFS (3.7 vs6.1 months; hazard ratio (HR) 2.12; *p* < 0.01) than patients receiving everolimus, while meidan overall survival (OS) was not significantly different but trended in favor of patients receiving everolimus (16.5 v 22.8 months; HR 1.77; *p* = 0.06) [92, 93]. However, GDC-0980 was reported to be well tolerated and to have early signs of anti-tumor activity in patients with advanced solid tumors or non-Hodgkin lymphoma, with an 80% decrease in measurable tumor marker [90]. A PhaseI/II study of GDC-0980 in patients with prostate cancer is ongoing.

In a phase Ib study of GDC-0980 in combination with capecitabine, 19 patients with advanced solid tumors and colorectal cancer were enrolled [94]. Confirmed partial responses (PR) were observed in one head and neck squamous cell cancer patient and one colorectal cancer patient with PIK3CA and KRAS mutations, which indicated preliminary anti-tumor activity of GDC-0980 in combination with capecitabine. GDC-0980 combined with fluoropyrimidine-based regimens was also demonstrated to be well tolerated, with confirmed antitumor activity [95].

#### PF-04691502 and PF-05212384 (Gedatolisib, PKI-587)

PF-04691502 and PF-05212384 (gedatolisib, PKI-587) are potent ATP competitive dual class-I PI3K/ mTOR kinases inhibitors. Preclinical studies demonstrated that PI3K-mTOR inhibition with PF-04691502 can enhance TP53/p73 expression and significantly inhibit tumor growth in head and neck squamous cell carcinomas [96]. In cancer cell lines with PI3Ka mutation and PTEN deletion, PF-04691502 can reduce phosphorylation of AKT and S6RP, thus inhibit cell proliferation [97]. PF-05212384 were reported to suppress a negative feedback loop mediated by mTORC2, leading to MEK/ERK over-activation in pancreatic cancer cells [98]. PF-05212384 causes strong attenuation of cell cycle and G0/G1 arrest, as well as induction of apoptosis in neuroendocrine tumor cells [99]. Phase I study of PF-04691502 in 23 patients with advanced solid tumors recommended that 8 mg orally once daily was tolerable, but objective anti-tumor responses were not observed in these patients [100]. The most frequent treatment-related AEs in the study population were fatigue, decreased appetite, nausea, hyperglycemia and rash. Maximum tolerated dose (MTD) for PF-05212384 was estimated to be 154 mg weekly in a phase II trial; the most common AEs were mucosal inflammation, stomatitis, nausea, decreased appetite, vomiting and fatigue [101]. Clinical benefits were noted in 11 of 78 patients, with 2 confirmed PR, 1 unconfirmed PR, and 8 long-lasting stable (> 6 months) [101].

A multi-arm phase I study evaluated dose-limiting toxicity, safety, pharmacokinetics and preliminary antitumor activity of the PF-04691502 and PF-05212384 plus irinotecan or the MEK inhibitor PD-0325901 in advanced cancer [102]. In this clinical study, MTD for PF-05212384 plus irinotecan (180 mg/m2) was estimated to be 110 mg weekly, and for PF-05212384 plus PD-0325901 (4 mg BID) was not reached at the highest dose at PF-05212384 154 mg weekly; the PF-04691502 (4 mg/6 mg, QD) combination arms were terminated early due to poor tolerability. Further preliminary evidence of clinical activity was observed in PF-05212384 combination arms. Similar results were also reported in a phase II study, which demonstrated poor tolerability of PF-04691502, Whilst also demonstrating acceptable tolerability and moderate anti-tumor activity of PF-05212384 in patients with recurrent endometrial cancer [103]. Ongoing clinical studies are exploring efficacy of PF-05212384 alone and in combination in breast cancer, lung cancer, head and neck cancer, ovary cancer, endometrial cancer, and pancreatic cancer.

### Pan-PI3K inhibitors

#### BKM120 (NVP-BKM120, Buparlisib)

BKM120 (buparlisib) is an orally pan-class I, reversible inhibitor of PI3K. In vitro, buparlisib demonstrates potent antiproliferative effect in human cancer cell lines. In vivo, buparlisib exhibits good oral bioavailability and significant antitumor activity in human tumor xenograft models at tolerated doses [104]. In the first-in-human, phase I, dose-escalation study of buparlisib in western patients with advanced solid tumors, MTD was established at 100 mg daily [105], which was confirmed in the dose-expansion part of another study [106]. The most common treatment-related AEs included rash, hyperglycemia, diarrhea, anorexia, mood alteration, decreased appetite, nausea and abnormal hepatic function [105, 106]. Phase I studies of buparlisib in Japanese and Chinese patients with advanced solid tumors also established a recommended dose of 100 mg daily [107, 108]. The MTD was 80 mg/d in a phase I study of buparlisib in patients with advanced acute leukemias [109].

A phase I trial in patients with advanced solid tumors suggested that the MTD of buparlisib in combination with standard doses of mFOLFOX6 (every 2 weeks of a 28-day cycle) was 40 mg daily; increased toxicity was observed compared to that expected from either buparlisib or mFOLFOX6 alone [110]. This trial concluded that further studies of buparlisib in combination with mFOLFOX6 are not recommended in gastrointestinal tumor. In a phase Ib clinical trial, addition of buparlisib (100 mg/day) to carboplatin + paclitaxel was well tolerated in patients with advanced solid tumors [111]. Confirmed objective response was observed in 5 of 25 patients with measurable disease, in particularly, all 3 patients with loss of PTEN expression benefitted clinically from treatment [111]. Interestingly, in the dose expansion study, this combination was revealed to show no significant clinical activity amongst the group of PTEN deficient tumors [112].

In combination with trametinib (MEK inhibitor), buparlisib 60 mg daily plus trametinib 1.5 mg daily displayed promising antitumor activity in patients with KRAS-mutant ovarian cancer, however, modest antitumor activity was observed in patients with non–small cell lung cancer and pancreatic cancer [113]. In a phase I dose escalation study, the MTD of combining buparlisib with olaparib (PARP inhibitor) was determined to be BKM120 50 mg daily and olaparib 300 mg daily. Anticancer activity was observed in patients with breast cancer and ovarian cancer [114]. However, in a phase II study, buparlisib was associated with a poor safety profile and minimal antitumor activity in advanced or recurrent endometrial carcinoma [115]. In patients with metastatic renal cell carcinoma progressing on vascular endothelial growth factor (VEGF) targeted therapies, buparlisib (80 mg/day) with bevacizumab (10 mg/kg every 2 weeks), was shown to be a tolerable regimen with preliminary activity [116]. In patients with castration-resistant prostate cancer, buparlisib did not demonstrate significant activity in a phase II trial, furthermore, the combination of buparlisib with abiraterone acetate was not recommended as a phase Ib study reported [86, 117].

Several clinical trials investigated the use of buparlisib in patients with breast cancer. The combination of buparlisib with capecitabine in patients with metastatic breast cancer was suggested to be well-tolerated in patients with metastatic breast cancer, with 5 of 17 patients demonstrating complete responses (CR) or PR [118]. The combination of buparlisib (100 mg/day) and trastuzumab (2 mg/kg every week) was well tolerated, and preliminary signs of antitumor activity were observed in patients with HER2-positive advanced breast cancer resistant to trastuzumab-based therapy [119]. A randomized adaptive phase II/III study (BELLE-4) suggested that addition of buparlisib to paclitaxel did not improve PFS of patients with HER2 negative advanced breast cancer [120]. In a placebo-controlled phase II trial (NeoPHOEBE), addition of the pan-PI3K inhibitor buparlisib to taxane-trastuzumab-based therapy in HER2 positive early breast cancer was revealed to be unfeasible [121].

Combination trials of buparlisib with endocrine therapy were conducted. MTD was estimated as buparlisib 100 mg daily plus fulvestrant in patients with metastatic estrogen receptor positive breast cancer in a phase I trial [122]. The most common AEs included fatigue, transaminases elevation, rash, and diarrhea. In a phase 3, randomized, placebo-controlled trial (BELLE-2), the addition of buparlisib to fulvestrant significantly prolonged PFS (6.9 vs.5.0 months, HR0.78, one-sided *p* = 0·00021) compared with the placebo plus fulvestrant group in postmenopausal women with hormone-receptor-positive, HER2-negative, advanced breast cancer [123]. Prespecified exploratory analyses in BELLE-2 showed that the combination regimen resulted in meaningful clinical benefits in the patients with circulating tumor DNA (ctDNA) PIK3CA mutant. Serious AEs were reported in 134 (23%) of 573 patients in the buparlisib group compared with 90 (16%) of 570 patients in the placebo group. Based on these findings, BELLE-3 was to assess the efficacy of buparlisib or placebo in combination with fulvestrant in hormone-receptor-positive, HER2-negative, advanced breast cancer patients with PIK3CA-mutant and wild-type status detected in ctDNA [124]. Buparlisib group was shown to have better PFS than the placebo group (3.9 vs.1.8 months, HR0.67, one-sided *p* = 0.00030), but serious AEs were more frequently reported in the buparlisib group (22% vs. 16%).

#### BAY 80–6946 (Copanlisib)

BAY 80–6946 (copanlisib) is an intravenous, potent, highly selective and reversible pan-class I PI3K inhibitor with predominant activity against the p110α and p110δ isoforms, currently in clinical development [125]. The first-in-human phase I study of copanlisib monotherapy in patients with advanced solid tumors and non-Hodgkin lymphomas determined the MTD to be 0.8 mg/kg (dosed intermittently on days 1, 8, and 15 of a 28-day cycle), and promising anti-tumor activity was observed, especially in patients with non-Hodgkin lymphoma [126]. The most common treatment-related AEs included nausea and transient hyperglycemia [126]. In a phase I study among Japanese patients with advanced or refractory solid tumor, MTD of 0.8 mg/kg was also observed; the most frequent AEs were hyperglycemia, hypertension, and constipation [127]. A phase I, dose-escalation study of copanlisib in combination with gemcitabine or cisplatin plus gemcitabine (CisGem) recommended copanlisib 0.8 mg/kg for patients with advanced cancer. Copanlisib plus CisGem demonstrated favorable clinical response than CisGem [128].

In a phase II study of copanlisib in different subtypes of indolent or aggressive lymphoma, the objective response rate was 44% (14/32) in indolent lymphoma and 27% (13/48) in the aggressive lymphoma. In this trial, enhanced antitumor effects were observed in tumors with upregulated PI3K pathway gene expression [129]. Based on this trial, another phase II trial was conducted with participants suffering from relapsed or refractory indolent B-cell lymphoma; overall response rates (ORR) of 59% (84/142) and CR rates of 12% were observed, leading to accelerated approval of copanlisib for relapsed follicular lymphoma [130, 131]. Clinical trials of copanlisib are ongoing, including several phase III trials in patients with non-Hodgkin lymphoma.

#### IPI-145 (Duvelisib)

IPI-145 (duvelisib) is an oral dual inhibitor of PI3K-δ and PI3K-γ currently in clinical development. Preclinical studies revealed that IPI-145 causes direct killing in primary chronic lymphocytic leukemia cells in a dose- and time-dependent manner, whereas not bring direct cytotoxicity to normal human B cells [132]. In a phase I, open-label study of duvelisib, the ORR in patients with relapsed/refractory peripheral T-cell lymphoma and cutaneous T-cell lymphoma were 50% (8/16) and 31.6% (6/19) respectively [133]. The most frequently reported AEs were transaminase increases, maculopapular rash, and neutropenia. Moreover, a phase II study is planned to further evaluate the efficacy and safety of duvelisib in patients with relapsed and refractory peripheral T-cell lymphoma. The samples of patients with chronic lymphocytic leukemia of this trial were obtained, and the gene-expression studies demonstrated that expression of anti-apoptotic protein BCL2 and several BH3-only pro-apoptotic genes were upregulated on duvelisib therapy [134]. In vitro, the combination of duvelisib and BCL2 inhibitor venetoclax resulted in enhanced apoptosis in chronic lymphocytic leukemia cells [134].

A phase I dose-escalation study in patients with relapsed/refractory indolent non-Hodgkin lymphoma reported the antitumor activity of duvelisib, with an ORR of 65% including CR in 25% of responding patients [135]. The phase II Dynamo study enrolled 129 patients with relapsed/refractory indolent non-Hodgkin lymphoma, and the ORR was 46%, with acceptable safety profile. The response rate across the disease subtypes was 41, 68, and 33% for patients with follicular lymphoma, small lymphocytic lymphoma, and marginal zone lymphoma, respectively [136]. More recently, in the randomized phase III DUO trial of duvelisib versus ofatumumab monotherapy, patients with relapsed or refractory chronic lymphocytic leukemia/small lymphocytic lymphoma were randomized to oral duvelisib 25 mg BID (*n* = 160) or ofatumumab intravenous (*n* = 159) [137]. Compared with ofatumumab group, patients who received duvelisib were shown to have significantly improving median PFS (13.3 months vs. 9.9 months; HR 0.52; *p* < 0.0001). The ORR was significantly higher with duvelisib (74% vs. 45%; p < 0.0001) regardless of del(17p) status. In September, 2018, the FDA granted regular approval to duvelisib for the treatment of adult patients with relapsed or refractory chronic lymphocytic leukemia or small lymphocytic lymphoma after at least two prior therapies. In addition, duvelisib received accelerated approval for adult relapsed or refractory follicular lymphoma patients who received at least two prior systemic therapies.

#### GDC-0941 (Pictilisib)

GDC-0941 (pictilisib) is a potent, orally class I pan-PI3K inhibitor, which is currently in clinical development [138, 139]. Pictilisib has demonstrated antitumor activity in human tumor xenograft murine models [140, 141]. Pictilisib exhibited favorable tolerability with potential clinical antitumor activity in the first-in-human phase I study of advanced solid tumor, and the MDT was 330 mg/day [142]. The most common drug-related toxicities were nausea, fatigue, diarrhea, vomiting, dysgeusia and decreased appetite [142]. Pictilisib demonstrated a favorable safety profile in Japanese patients with advanced solid tumor or non-squamous non-small cell lung cancer in a phase Ia/Ib study; no objective anti-tumor responses were observed in patients with advanced solid tumor while partial anti-tumor responses were observed in patients with non-squamous non-small cell lung cancer [143]. The MDT was determined to be 340 mg/day for monotherapy and was 260 mg/day for combination with carboplatin-paclitaxel and bevacizumab [143]. In patients with advanced solid tumors, another phase I dose-escalation study indicated that combination of pictilisib with EGFR tyrosine kinase inhibitor erlotinib was feasible [144]. In this study, modest antitumor effects were observed, that 2 (3.5%) of 57 patients experienced PR and 19 (33.3%) had stable disease [144]. A phase Ib dose-escalation study in patients with advanced non-small cell lung cancer assessed the tolerability and pharmacokinetics of pictilisib in combination with eitherpaclitaxel and carboplatin or pemetrexed and cisplatin, with or without bevacizumab [145]. In this study, pictilisib combination with various treatment regimens demonstrated promising efficacy and manageable toxicity, and preliminary antitumor activity was observed [145].

In a randomized, double-blind, placebo-controlled phase II study (FERGI) of oestrogen receptor-positive, aromatase inhibitor resistant advanced breast cancer, patients were randomly allocated (1:1 in part 1 and 2:1 in part 2) to pictilisib (340 mg daily in part 1 and 260 mg daily in part 2) or placebo, plus intramuscular fulvestrant 500 mg. As a result, the addition of pictilisib to fulvestrant did not significantly improve PFS; it may be that the dose of pictilisib was limited by toxicity, potentially limiting its efficacy [146]. A phase II randomized PEGGY study in patients with hormone receptor-positive, HER2-negative, locally recurrent, or metastatic breast cancer revealed that adding pictilisib to paclitaxel did not prolong PFS of the patients [147]. In a randomized phase II study, patients with newly diagnosed estrogen receptor–positive, HER2 negative breast cancers were randomized to anastrozole or pictilisib plus anastrozole group [148]. The antitumor effects were measured by change of Ki-67 protein expression between tumor legions taken before and at the end of treatment [148]. Patients receiving the combination therapy showed greater geometric mean Ki-67 suppression from 66.0 to 83.8%. Further, significant Ki-67 response was observed for patients with luminal B tumor, but not for patients with luminal A tumor [148].

#### GDC-0032 (Taselisib)

GDC-0032 (taselisib) is a potent and selective inhibitor of p110α, p110δ, and p110γ isoforms of class IA PI3K, with 31 folds less potency for the p110b isoform. Taselisib was progressed to clinical trials as a potential treatment for human cancer. A phase I study in Japanese patients showed that taselisib was well tolerated at 6 mg daily in patients with advanced solid tumor, and 4 mg daily in combination with fulvestrant in patients with HR-positive, HER2-negative advanced/recurrent breast cancer [149]. The most frequent treatment-related AEs were rash, diarrhea, and stomatitis. PR were observed in 2/9 patients receiving monotherapy, and in 1/6 patients receiving combination therapy [149]. All patients with PR had PIK3CA-mutated tumor, which suggested that taselisib is expected to be effective in patients with PIK3CA-mutated solid tumor [149]. In another phase I dose escalation study of taselisib, 34 patients with locally advanced or metastatic solid tumor were given 3–16 mg taselisib once daily [150]. Dose limiting toxicities (DLT) were observed in patients receiving 12 and 16 mg dose levels. Pharmacodynamic findings of patient tumor sample showed that PI3K pathway was inhibited at dose ≥3 mg/d. Confirmed response was observed in 5/14 of PIK3CA-mutant tumor patients, and in 0/15 patients with tumors without known PIK3CA mutations [150]. A randomized phase III study of taselisib plus fulvestrant versus placebo plus fulvestrant in patients with metastatic breast cancer is ongoing.

### Isoform-specific inhibitors

#### BYL719 (Alpelisib)

BYL719 (alpelisib), an oral selective PI3Kα isoform inhibitor, exhibited dose-dependent antitumor activity in tumor xenograft models, particularly models with mutated or amplified PIK3CA, highlighting the potential antitumor activity of alpelisib in patients with PIK3CA-altered tumors [151, 152]. The first-in-human phase Ia study of alpelisib, demonstrated a tolerable safety profile and declared its MTD as 400 mg daily and 150 mg twice daily [153]. The most frequent treatment-related AEs included hyperglycemia, nausea, decreased appetite, diarrhea, and vomiting [153]. Among 134 patients with PIK3CA-altered advanced solid tumor who received treatment, stable disease was achieved in 70 (52.2%) patients, PR was achieved in 7 (5.2%) patients, and CR was achieved in 1 (0.7%) patient [153]. In patients with ER-positive, HER2-negative metastatic breast cancer refractory to endocrine therapy, MTD of alpelisib in combination with letrozole was 300 mg/d [154]. In this phase Ib study, the clinical antitumor activity was observed in 44% patients with PIK3CA mutated and 20% in PIK3CA wild-type tumors [154]. In trastuzumab- and taxane-resistant HER2-positive metastatic breast cancer, the combination of alpelisib and trastuzumab emtansine was tolerable and activity was observed, therefore further studies of the combination are expected to perform [155]. The triple-combination therapy of encorafenib (RAF kinase inhibitor), cetuximab (monoclonal antibody targeting EGFR) and alpelisib demonstrated promising clinical activity and tolerability in metastatic BRAF-mutant colorectal cancer patients [156]. A phase III study of alpelisib and fulvestrant is ongoing.

#### CAL-101 (GS-1101, Idelalisib)

CAL-101 (GS-1101, idelalisib) is an oral and specific inhibitor of the δ isoform of PI3K [122, 123]. It has been shown that idelalisib has therapeutic effects without inhibiting PI3K signaling essential for normal function of healthy cells [157, 158]. Idelalisib is the frst FDA-approved PI3K inhibitor for use in combination with rituximab for the treatment of relapsed or refractory chronic lymphocytic leukemia, or as monotherapy for relapsed small lymphocytic lymphoma and follicular lymphoma previously treated with two or more prior systemic therapies.

In a phase Ib dose-escalation and extension studies of idelalisib, 64 patients with relapsed/refractory B-cell malignancies were assigned to one of eight regimens; idelalisib was taken once or twice a day at doses ranging from 50 to 350 mg [159]. The ORR was 47% (30/64), with 1 patient had a CR (1.6%). The median duration of response was 18.4 months, and the PFS was 7.6 months [159]. AEs were reported in 20% or more patients, including diarrhea, fatigue, nausea, and rash [159]. In this 48-week phase I clinical trial, the results of 40 patients with relapsed/refractory mantle cell lymphoma were reported in another article. Among this population, it was reported that the ORR was 40% (16/40), with CR in 5% (2/40) patients. The median duration of response was 2.7 months, and the median PFS was 3.7 month [160]. In patients with relapsed/refractory chronic lymphocytic leukemia, acceptable safety profile and antitumor activity of idelalisib were also reported [161]. A phase II trial in patients with chronic lymphocytic leukemia found that idelalisib used as upfront therapy caused an early, severe hepatotoxicity, particularly in younger subjects who have not received prior disease-specific therapy [162]. A single-group, open-label, phase II trial evaluating patients with relapsed (after receipt of rituximab and an alkylating agent) indolent non-Hodgkin lymphomas demonstrated similar findings; 125 patients were administered idelalisib 150 mg twice daily [157]. The ORR was 57% (71/125), and 6% (7/125) met the criteria for CR, leading to FDA approval [9, 157, 163]. The median duration of response was 12.5 months, and the median PFS was 11 months [157]. Moreover, in patients with relapsed/refractory classical Hodgkin lymphoma, idelalisib was tolerable and had modest single-agent activity, with an ORR of 20% (5/25) [164].

The safety and efficacy of combined therapy with idelalisib and rituximab was evaluated in several clinical trials. In a phase II study of idelalisib plus rituximab, 64 treatment-naive older patients with chronic lymphocytic leukemia received rituximab 375 mg/m^2^ weekly and idelalisib 150 mg twice daily; the ORR was 97% (62/64), including 19% (12/64) CR [165]. Notably, the ORR was 100% in patients with del(17p)/TP53 mutations. As compared with placebo and rituximab, this combined treatment significantly improved ORR (81% vs. 13%; OR, 29.92; *P* < 0.001), PFS (HR, 0.15; P < 0.001), and OS at 12 months (92% vs. 80%; HR, 0.28; *P* = 0.02) among chronic lymphocytic leukemia patients who are less able to undergo standard chemotherapy [166]. However, the combination of idelalisib, lenalidomide and rituximab were not recommended for that excessively toxicity of this triplet regimen was reported in patients with relapsed and refractory lymphoma in a phase I trial [163]. In a global, randomised, phase III trial, idelalisib plus atumumab (a second-generation anti-CD20 antibody) resulted in better PFS (16.3 months vs.8.0 months, HR 0·27, *p* < 0·0001) compared with atumumab alone in patients with relapsed chronic lymphocytic leukaemia progressing less than 24 months from the last therapy [167].

## Resistances

The complexity of the PI3K/AKT/mTOR signaling network involves numerous feedback loops, extensive crosstalk nodes with other signaling pathways and compensatory pathways, providing ample opportunities for circumventing the effects of PI3K inhibition. Although small-molecule inhibitors of PI3K have exhibited promising clinical efficacy against human cancers, intrinsic and acquired resistance limits their therapeutic efficacy. Therefore, elucidating the mechanisms underlying resistance to PI3K inhibitor can provide rationale for combination therapies and alternative therapies. The specific mechanism is not completely defined; however, recent studies have described several possible resistance mechanisms, including PI3K reactivation, activation of parallel pathway, and tumor microenvironment.

Acquired amplification and mutation of PIK3CA and PIK3CB, which resulted in a marked upregulation of the PI3K signaling itself, have been shown to cause resistance to selective PI3K inhibitors [168, 169]. As suggested previously, in the absence of PTEN, proliferation of cancer cells became dependent mostly on the activity of the p110β isoform [170, 171]. The impact of PTEN loss on PI3Kα inhibitor resistance has been proposed [172]. The loss of PTEN alone was not able to induce resistance to inhibitor of class I PI3K (GDC-0941), however, amphiregulin enhanced the resistance, which resulted in increased EGFR/MAPK signaling. As a PI3K regulatory subunit, the phosphorylation of p85 has also been suggested to play a role in the development of resistance to PI3K inhibitors; presence of a regulatory loop between PI3K p85 and Src has also suggested contributing to resistance against PI3K inhibitors [173]. Intrinsic resistance to PI3K p110a Inhibitors was correlated with sustained mTORC1 activity; growth factors such as insulin-like growth factor 1 and neuregulin 1 can activate mTOR and thus mediate resistance to p110a inhibitors [152].

The RAS-RAF-MEK-ERK signaling pathway is highly interconnected with PI3K signaling [174]. Mutation and overexpression of HRAS which belongs to the RAS family has been shown to reduced susceptibility to PI3K inhibitor, while knockdown improved sensitivity [175]. Further, interactions between NEK9 and MAP2K4 have been proposed to mediate cancer cell proliferation and resistance to PI3K inhibitors [176]. PI3K inhibition with the pan-PI3K inhibitor GDC0941/ XL-147 or the dual PI3K/mTOR inhibitor BEZ235 has been shown to induce increased HER2/3 expression and lead to compensatory activation of the ERK signaling pathway [177, 178]. Activation of STAT5 and expression of Pim kinases through STAT5 also conferred resistance to PI3K/AKT inhibitors by enhancing the mTORC1/Mcl-1 pathway [179]. Dual inhibition of PI3K and m-TOR has been found to elicit a positive feedback response and lead to increases activation of JAK2/STAT5 and secretion of IL-8, thus contributing to drug resistance [180]. Moreover, IL6-STAT3 loop triggered epithelial–mesenchymal transition and expanded action cancer stem cells population, which have been proposed as one of the mechanisms [181]. Aberrant regulation of WNT/β-catenin signaling and activation of GSK3β were correlated with resistance to the dual PI3K/mTOR inhibitor; nuclear β-catenin conferred resistance to the FOXO3a-mediated apoptosis provoked by PI3K and AKT inhibitors [182, 183].

Dual PI3K/mTOR inhibition led to activation of the NOTCH-MYC pathway [184]. NOTCH pathway and downstream induction of c-MYC were conferred resistance to PI3K inhibitors, whereas overexpression of the NOTCH canonical target genes HES1, HEY1 or HEY2 were not correlated with PI3K pathway inhibitor resistance [37, 184, 185]. The MYC was involved in growth, proliferation, differentiation, and metabolism of malignant cells, and knockdown of MYC reversed the resistance to dual PI3K/mTOR inhibitor [184]. Previous studies have also indicated that amplification of both MYC and eIF4E can mediate resistance to PI3K/m-TOR inhibitors [186]. eIF4E is an established MYC regulated target, indicate that interactions between MYC and eIF4E in regulating resistance mechanism is a possibility [184].

Proviral Integration site for Moloney murine leukemic virus (PIM) which overexpress in multiple malignancies has been shown to confer resistance by maintaining activation of downstream PI3K effectors in an AKT-independent manner [187]. In addition, PIM has been reported to modulate the activity of eIF4B and mTORC1 to enhance NRF2/ARE activity, and to decrease ROS production to diminish the cytotoxicity of PI3K/AKT inhibitors [188]. S-phase kinase-associated protein 2 (Skp2) could promote the activation of AKT, and it has been reported to correlate with the resistance of PI3K inhibition [189]. Amplification or overexpression of RSK3 (Ribosomal S6 kinases RPS6KA2), RSK4 ((Ribosomal S6 kinases RPS6KA4), PAK1, CDK 4/6, MSK1 (mitogen- and stress-activated protein kinase 1), KDM6B, and IGFBP5 have also been shown to confer resistance to PI3K inhibitors [168, 190–192].

High amounts of purine-related aqueous metabolites like hypoxanthine, and high levels of the mRNA encoding hypoxanthine phosphoribosyl transferase 1 (one of the key components of the purine salvage pathway), have been found to be associated with resistance of PI3K pathway inhibition [193]. In consideration of the fact that ncRNA have been reported to regulate PI3K signaling and other parallel pathways (e.g. WNT/β-catenin, RAS/ERK/MAPK, JAK/STAT, NOTCH), we believe ncRNA may also play a role in the resistance of PI3K inhibitors [194–199]. Not surprisingly, more and more researches have suggested that deviant ncRNA expression is powerfully concerned about tumor drug resistance [200–208]. Recent studies have indicated potential mechanism of acquired resistance to dual PI3K/mTOR inhibitors, including elevated glycolysis accompanied with depletion of mitochondrial DNA, and upregulated DNA methyltransferases which Reduce PTEN and PPP2R2B expression [209, 210]. Novel roles of the tumor microenvironment have introduced in regulating drug resistance, and macrophages in microenvironment have been proposed as factors contributing to the resistances of PI3K inhibitors through the activation of NF-κB signaling [211].

## Conclusions

The PI3K signaling pathway plays an important role in cell growth, proliferation and survival, making PI3K inhibition an attractive target for anticancer therapy. However, clinical trials with PI3K inhibitors used as a monotherapy have shown limited clinical activity, possibly as a consequence of resistance to PI3K inhibition and poor tolerability of PI3K inhibitors. Dual PI3K/ mTOR and pan-PI3K inhibitors have made their way into clinical trials with limited efficacy as monotherapy, and relatively high rates of side effects were reported. As it has been increasingly recognized that different isoforms of PI3K play non-redundant roles in particular tumor types, isoform-selective inhibitors were developed. Isoform-selective PI3K inhibitors demonstrate improved specificity and reduced toxicity over dual PI3K/ mTOR and pan-PI3K inhibitors, which have shown promising success in several clinical trials for both solid and hematological malignancies.

Several studies showed that PI3K inhibitors were more effective in patients with PI3K pathway mutations, however, some patients without documented PI3K mutations benefited from PI3K inhibitors and some patients with PIK3CA or other mutations not experienced benefit. As a result, strong correlations between PI3K mutations and response to therapy still have not been established in preclinical and clinical studies. It is important to identify reliable biomarkers that can guide patient selection, and to determine which tumor type and genetic profiles will benefit from PI3K inhibition. It is reported the value of pharmacodynamic biomarkers and functional imaging monitoring biomarker in guiding the selection of patients who are most likely to respond to PI3K inhibition, but the precision is still controversial [212]. To date, the mechanism of PI3K inhibitors has not been well established. The precise mechanism needs to be extensively and systematically studied, so that it will allow us to monitor efficacy and side effects, and to make personalized therapeutic decisions.

Preliminary clinical data indicated that the use of single-agent PI3K pathway inhibitors achieved modest responses and was unlikely to be a curative therapy for diverse cancers. The efficacy of PI3K inhibitors is limited for their narrow therapeutic window and frequent treatment-related toxicities. The drugs recommended are more likely to be optimally used in combination with other therapeutic modalities, such as surgery, hormonal therapies and other anticancer agents. Introduction of tumor suppressive or knockdown of oncogenic ncRNAs would be a feasible approach to inhibit the PI3K pathway. The combination of PI3K inhibitors with ncRNAs or inhibitors against other cross-talk pathways might yield promising therapeutic effects. AEs, including nausea, vomiting, diarrhea, hyperglycemia, fatigue, rash, anorexia, and abnormal hepatic function were frequently reported. These combination strategies may also decrease the rates of AEs and minimize the risk of the development of resistance.

Overall, PI3K inhibition is being investigated as a potential strategy to develop novel therapeutics for cancer management. Although we move forward with the clinical development of PI3K inhibitors, maximizing the utility of these agents in the treatment of patients remains challenging. Certainly, understanding the precise mechanisms of PI3K signaling and PI3K inhibition will be critical. Optimization of the patient selection strategies and combination approaches will help increase the practical efficacy of these agents. Continued work to clarify the resistance mechanisms and the novel strategies to overcome resistance will also be important.

## Abbreviations

AEs: Adverse events
CR: Complete responses
ctDNA: Circulating tumor DNA
FDA: Food and Drug Administration
HR: Hazard ratio
LncRNA: Long non-coding RNA
miRNA: MicroRNA
MTD: Maximum tolerated dose
mTOR: Mammalian target of rapamycin
ncRNA: Non-coding RNA
ORR: Overall response rates
OS: Overall survival
PFS: Progression-free survival
PI3K: Phosphatidylinositol-3-kinase
PIP2: Phosphorylation of PtdIns(4,5) P2
PIP3: PtdIns(3,4,5) P3
PR: Partial responses
PTEN: Phosphatase and tensin homologue deleted on chromosome 10
RDE: Recommended dose for expansion
